# Novel 1, 2, 4-Triazoles as Antifungal Agents

**DOI:** 10.1155/2022/4584846

**Published:** 2022-03-22

**Authors:** Zahra Kazeminejad, Mahrokh Marzi, Abolfazl Shiroudi, Seyed Amin Kouhpayeh, Mojtaba Farjam, Elham Zarenezhad

**Affiliations:** ^1^Young Researchers and Elite Club, Tonekabon Branch, Islamic Azad University, Tonekabon, Iran; ^2^Noncommunicable Diseases Research Center, Fasa University of Medical Sciences, Fasa, Iran; ^3^Young Researchers and Elite Club, East Tehran Branch, Islamic Azad University, Tehran, Iran; ^4^Department of Medical Pharmacology, School of Medicine, Fasa University of Medical Sciences, Fasa, Iran

## Abstract

The development of innovative antifungal agents is essential. Some fungicidal agents are no longer effective due to resistance development, various side effects, and high toxicity. Therefore, the synthesis and development of some new antifungal agents are necessary. 1,2,4-Triazole is one of the most essential pharmacophore systems between five-membered heterocycles. The structure-activity relationship (SAR) of this nitrogen-containing heterocyclic compound showed potential antifungal activity. The 1,2,4-triazole core is present as the nucleus in a variety of antifungal drug categories. The most potent and broad activity of triazoles have confirmed them as pharmacologically significant moieties. The goal of this review is to highlight recent developments in the synthesis and SAR study of 1,2,4-triazole as a potential fungicidal compound. In this study, we provide the results of a biological activity evaluation using various structures and figures. Literature investigation showed that 1, 2, 4-triazole derivatives reveal the extensive span of antifungal activity. This review will assist researchers in the development of new potential antifungal drug candidates with high effectiveness and selectivity.

## 1. Introduction

Heterocyclic organic chemistry is a main field in organic and medicinal chemistry [1–4]. Azoles are *nitrogen-*containing five-membered heterocyclic compounds [5, 6]. The presence of nitrogen in heterocycles has a major effect on biological activity. Recently, azole compounds have become hot topics around the world [2, 7]. Among the azoles fused as heterocyclic compounds, 1,2,4-triazole derivatives with molecular formula (C_2_H_3_N_3_) are the most stable compounds [8]. 1,2,4-Triazoles showed broad ranges of biological activities, such as antimalarial [9], antiurease [10], antiviral [11], anticonvulsant [12], antioxidant [13], and antifungal [14]. Some of the medicinal plants containing triazole scaffolds were demonstrated to be antifungal agents, including cyproconazole, triadimefon, metconazole, tebuconazole, propiconazole, epoxiconazole, and prothioconazole [15]. Annually, invasive fungal infections cause 1.7 million deaths in the world, which is a major public health issue [16]. One of the most serious issues is the rise of synthetic drug resistance to various fungal pathogens; thus, the synthesis and development of new 1,2,4-triazoles with low toxicity are essential worldwide [17]. This group of bioactive compounds acts by inhibiting the activity of cytochrome P450-dependent enzyme, the lanosterol 14*α*-demethylase (CYP51), which is an important enzyme in fungi ergosterol biosynthesis [18]. Azoles link to the iron in porphyrins, causing a blockade of the fungal ergosterol biosynthesis pathway resulting in the agglomeration of 14-demethylated sterols [19]. Recently, novel derivatives of 1,2,4-triazoles were prepared and evaluated for fungicidal activity and some of them showed potential activity against certain fungi. In previous years, many research articles have emphasized the importance of 1,2,4-triazoles as potent antifungal and antibacterial properties [20–31]. However, this review is focused on the latest papers (2015–2021) in the synthesis of new 1,2,4-triazole as an antifungal agent and evaluating structure-activity relationship (SAR) to provide an insight for the logical synthesis of more effective 1,2,4-triazole antifungal candidates. The diagram of choosing publications and the content of this review are illustrated in Figure 1.

## 2. Synthesis of 1,2,4-Triazoles

1,2,4-Triazoles are five-membered sp^2^ hybridization compounds containing three nitrogen atoms at the 1-, 2-, and 4-positions of the ring. There are two tautomeric forms: 4*H*-1,2,4-triazole and 1*H*-1,2,4-triazole (Scheme 1) [32].

### 2.1. General Pathways

A simple method for preparing 1,2,4-triazoles has been introduced from the reaction of formamide and hydrazines without a catalyst using microwave irradiation (Scheme 2) [33].

A series of 1,3-disubstituted-1,2,4-triazoles were synthesized by reacting amidine and trialkyl amines with K_3_PO_4_ as a base in the presence of a copper (II) catalyst (Scheme 3) [34].

I_2_-mediated oxidative N-S and C-N bond formations are an ecologically friendly and effective approach for synthesizing novel 1,2,4-triazoles from isothiocyanates (Scheme 4) [35].

1,5-Disubstituted-1,2,4-triazoles were prepared using copper (II) as the catalyst. This regioselective method makes it simple to produce 1,2,4-triazole moiety with wide substrate amplitude, high yield, and significant functional group compatibility (Scheme 5) [36].

The synthesis of 1,2,4-triazoles from aliphatic amines and hydrazones has been developed using a cascade C-H functionalization, oxidative aromatization sequence, and double C-N bond formation under iodine as the catalyst (Scheme 6) [37].

### 2.2. Synthesis by Substitution of 1,2,4-Triazole

#### 2.2.1. Arylation Reactions

Under reflux circumstances in pyridine, 1-aryl-1,2,4-1*H*-triazole is arylated by an aryl halide with electron-withdrawing groups using CuO as the catalyst (Scheme 7) [38, 39].

#### 2.2.2. Alkylation

When sodium methoxide in methanol is used as the base, 1,2,4-triazole is alkylated at the *N*1 position, yielding in a mixture of 1-methyl- and 4-methyl-1,2,4-triazole with methyl sulfate alkylation in NaOH (Scheme 8) [40].

### 2.3. Direct the Synthesis of *N*4-Substituted Triazoles

A group of 4-Arylsubstituted-1,2,4-4*H*-triazoles yields via the reaction of *N*, *N*-diformylhydrazine with primary amine at high temperatures (Scheme 9) [41]. Pellizzari and Soldi pioneered this system by reacting simple arylamines such as naphthylamine, aniline, or toluidine with *N*, *N*′-diformylhydrazine [42, 43], as well as downloading via slight changes in amino heterocycles containing 3-amino-1,2,4-4*H*-triazole to generate 3,4-bitriazoles [44–46].

## 3. Pharmaceutical Drugs

### 3.1. Chemical Structures of 1, 2, 4-Triazole-Based Marketed Drugs

Bladin were the first to synthesize 1,2,4-triazoles in 1885 [31]. The primary procedures, such as the reaction of formamide with formylhydrazine, produced low yields of 1,2,4-triazole [47, 48]. Later, it was found that condensation of formamide with hydrazine sulfate yielded 1,2,4-triazole in average yield. Various pharmacological activities of 1,2,4-triazoles as antifungal [42, 49, 50] have been observed which included fluconazole, isavuconazole, itraconazole, voriconazole, ravuconazole, and posaconazole (Figure 2). Several 1,2,4-triazole-based drugs are under clinical use for the treatment of different diseases. Some of the most effective drugs available in the market are described in the following Table 1.

### 3.2. Structure-Activity Relationship of Fluconazole

Fluconazole is well known as one of the most potent antifungal drugs with remarkable interest in medicinal chemistry. Due to the importance of fluconazole as a reference drug, the structure-activity relationship is shown in Figure 3.

## 4. 1,2,4 Triazole Scaffold for the Development of Antifungal Agents

This part of the review is classified into two parts based on the structural similarities of 1,2,4-triazole derivatives. First, we explained novel analogues of commercial 1,2,4-triazole drugs and then discussed 1,2,4-triazole-based scaffolds with various functional groups such as indole, benzimidazole, quinolone, quinazoline, amine, hydrazone, amide, sulfur, and oxime ether that showed remarkable antifungal properties, as well as SARs of all synthesized compounds.

### 4.1. Analogues of Commercial 1,2,4-Triazole Drugs

Most triazole compounds containing 1,2,3-benzotriazine-4-one demonstrated more antifungal activity against *Candida albicans* and *Cryptococcus neoformans* than reference drug with MIC values ranging from 0.0156 to 2.0 *μ*g/mL. Furthermore, a strong SAR investigation revealed that derivatives with groups −NO_2_ and CF_3_ at the 7-position exhibited more effective antifungal activity than derivatives with groups at the 5-, 6-, and 8-positions. In addition, products containing halogens such as Cl and F demonstrated more excellent antifungal activity than those containing electron-withdrawing groups. Meanwhile, compound 1a (R = 7Cl) demonstrated remarkable antifungal activity specifically against *Aspergillus fumigatus* (MIC = 0.25 *μ*g/mL) and moderate activity against fluconazole-resistant *Candida albicans* strains (Figure 4) [88].

Blokhina et al. [29] investigated the fungicidal activity of thiazolo[4,5-*d*] pyrimidine hybrids with (1*H-*1,2,4) triazole. All derivatives include the methyl-(2a), fluoro-(2b), and chloro-(2c) substituents at the *para* position. *In vitro* evaluation of various compounds with a potent alkylpiperazinyl linker demonstrated antifungal activity similar to the standard drug. The most active compounds are methyl-(2a), fluoro-(2b), chloro-(2c) methyl-(3a), and fluoro-(3b). Based on MIC values, antifungal activity is classified as poor (≥32 *μ*g/mL), modest (16–32 *μ*g/mL), good (4–8 *μ*g/mL), excellent (0.06–2 *μ*g/mL), or outstanding based on MIC values (Figure 5).

Montoir et al. [89] reported a novel class of azole antifungal compounds based on a pyrrolotriazinone scaffold. As a result, these compounds demonstrated fungicidal activity against pathogenic Candida species *in vitro* (fluconazole susceptible and fluconazole resistant) and were more active than voriconazole against two Candida *albicans candidates*. Compound 4e also showed promising *in vitro* activity against several filamentous fungi, including *Aspergillus fumigatus* (Figure 6).

Xie et al. [90] demonstrated that the entire series of triazole containing isoxazole compounds (5a-f) were antifungal against eight human pathogenic fungi. Compound 5a showed a strong inhibitory activity toward *Candida parasilosis* and *Candida albicans* with MIC80 values of 0.0313 *μ*g/mL. According to the SARs study, mono-fluorine on the phenyl ring possesses antifungal activity. On the other hand, enhancing the number of fluorine atoms (5c-d) may result in a reduction in antifungal activity (Figure 7).

In comparison to the reference drugs, voriconazole, fluconazole, and ravuconazole, an alkyne linked in the side chain of the triazole derivatives demonstrated good fungicidal activity against eight human pathogenic fungi, with particularly noticeable activity against Cryptococcus species and Candida. Compounds 6b and 6c shown *in vitro* antifungal activity against all the investigated fungi with (MIC80 = 0.0156–0.5 mg/mL), which is greater than fluconazole and ravuconazole. SAR study shows that *para* fluoro (6e, 6h), *para* chloro (6b), and *para* cyano (6c) substituted phenylalkynyl, or pyridinyl alkynyl (6m, 6n) side chains improve activity. Compounds with R groups in the *para* position are shown to be more active than *meta* or *ortho* compounds (Figure 8) [91].

The antifungal efficacy of triazole alcohol derivatives toward 16 *Candida* isolates from five different species, including fluconazole-susceptible and fluconazole-resistant isolates, was investigated. All of these derivatives with MIC values of 0.063–1 mg/mL showed higher activity than fluconazole (MICs = 0.5–4 mg/mL) against fluconazole-susceptible isolates; significantly, compounds 7b and 7e were also active against fluconazole-resistant species. However, the effect of chloro substitution depends on the type of species. For example, the 2,4-dichloro substituent 7d was shown to be more effective against *C. albicans* than 3-Cl (7b) or 4-Cl (7c). In the case of *C. krusei*, however, the 3-chloro group was better than the 4-chloro or 2,4-dichloro substituents. The addition of fluoro or bromo groups to the benzyl residue, however, had no beneficial impact. Among the fluorobenzyl regioisomers (7f-h), the 3-fluoro 7g analog was more active against *Candida* species (Figure 9) [92].

Chandrika et al. [93] investigated novel fluconazole (FLC) compounds for antifungal activity against the clinical strains of *C. parapsilosis*, *C. glabrata*, and *Candida* with aryl, alkyl, cycloalkyl, and dialkyl-amino substituents for neoformans using MIC determination. The activity of the alkylamino FLC derivatives was shown to be directionally related to the length of the alkyl chains (Figure 10).

Tekale et al. [94] investigated the antifungal activities of triazole compounds, including imidazole. The impact of the imidazole side chain on the *in vitro* fungicidal activity of novel synthesized compounds toward various microorganisms such as *aspergillus*, *niger*, *aspergillus fumigates*, and *Candida albicans* was demonstrated. Compound 9e had the lowest activity against *C. albicans*, and compounds 9b & 9d had higher activity against *A. niger* than the other compounds (Figure 11).

The MIC_80_ values of new triazole compounds containing 1,2,3-triazoles or substituted amines as side chain 10a-o derivatives demonstrated better antifungal properties than those of fluconazole on three significant fungal infections except for 10i. Furthermore, the considerable compounds 10d, 10 k, 10n, 10 m, and 10o were reported on the *Aspergillus fumigatus* strain (MIC_80_ range: 0.125–1 *μ*g/mL). In addition, 10k can be applied to almost all fungi tested, especially *Aspergillus* spp. In vitro biological assessments of the compounds 10d and 10k showed potent antifungal properties (Figure 12) [95].

Sadeghpour et al. [96] reported two classes of novel fluconazole-derivatives containing nitrotriazole or 2-(piperazin-1-yl) ethanol moieties, which were evaluated for antifungal activity against standards and clinically isolated yeasts, and their MIC structures were compared with those of fluconazole. Nitrotriazole derivatives 11a-d and compounds 12g and 11b containing two chlorine atoms exhibited good activity against the tested fungus, notably some fluconazole-resistant species. Compounds 11a, 11b, and 12g with 2,4-difluorophenyl or 2,4-dichlorophenyl groups had more excellent antifungal activity (Figure 13).

*In vitro* antifungal activities of new triazole derivatives of ravuconazole and isavuconazole were demonstrated against eight fungal isolates. Compounds 13e (2-F), 13f (2, 3-diF), and 13g (2, 4-diF) in particular displayed activity to ravuconazole, demonstrating that the 2,4-diflourophenyl group is more active than the 2,5-diflourophenyl group. Compounds without a fluoro substitution on the phenyl ring, such as 13a (4-CH_3_), 13c (4-SO_2_-CH_3_), 13b (4-NO_2_), and 13d (4-CN), were less active than those with fluorophenyl groups, such as 13k (2, 6-diF),13h (2, 5-diF), and 13l (2, 4, 6-triF) (Figure 14) [97].

Chen et al. [98] investigated a class of novel antifungal triazoles, and compound 14l (MIC = 0.125 *μ*g/mL) showed greater antifungal activity versus *Candida glabrata* and *Candida albicans*. Furthermore, compounds 14j, 14k, 14l, 15a, and 15b (MIC = 0.125–0.5 *μ*g/mL) were shown to be more effective than fluconazole (MIC = 0.25 *μ*g/mL) against *C. glabrata*. SARs revealed that 3-substitutions (14d, 14e, and 14f) were more favorable than the 4-substitutions (14b, 14c), while electron-rich thiophene (14h, 14i) significantly outperformed the electron-deficient pridinyl group in antifungal activity (14g). Antifungal activity may be enhanced by replacement of the phenyl group of compound 14a by a cycloalkyl group, namely, cyclopentyl (14j), cyclohexyl (14k), and cyclopropyl (7l). In contrast, *tert-butyl* substitution (14m) only showed modest activity (Figure 15).

Compared to fluconazole and 5-flucytosine, the new fungicidal hybrids of 5-flucytosine and fluconazole showed modest antifungal activity. Surprisingly, a hybrid of 3,4-dichlorobenzene can inhibit clinical-resistant strain *C. albicans* and the growth of *C*. *albicans* ATCC 90023 with MIC values of 0.02 and 0.008 mM, respectively. Compound 16e inhibited *C. albicans* rapidly, whereas compound 16a lacked fungicidal activity due to the lack of substituents on the phenyl ring (ure 16) [99].

Xu et al. [100] described a series of novel triazole derivatives having *γ*-lactam that were screened for antifungal activity against six pathogenic fungi *in vitro*. Furthermore, the pyridyl- and phenyl-substituted compounds 17d and 17e showed moderate antimicrobial activity against *Cryptococcus neoformans* and *Candida* spp. (Figure 17).

Zhang et al. [101] reported the triazole sequence as a miconazole analogue with antifungal against five fungi. Among these compounds, 18b, 3,4-dichlorobenzyl had the highest activity. Furthermore, the antifungal activity of 3,4-dichlorobenzyl compound 18b (MIC = 0.5 *μ*g/mL), 2,4-difluorobenzyl derivative 18c (MIC = 4 *μ*g/mL), and 2-fluorobenzyl miconazole analogue 18e (MIC = 16 *μ*g/mL) due to F or Cl may be significantly improved over nitro group compound 18d (nitrobenzyl). Surprisingly, substituted benzyl triazoles (MIC = 0.5–16 *μ*g/mL) showed more potency than monosubstituted benzyl compounds (MIC = 0.5–32 *μ*g/mL) (Figure 18).

The antifungal activity of a novel triazole-piperdine-oxadiazoleside group against clinically important fungal pathogens was investigated. Particularly, 19g (MIC = 0.031 *μ*g/mL) and 20b (MIC = 0.016 *μ*g/mL) showed high activity versus *Candida albicans* including fluconazole-resistant strains. Compounds 19c, 19d, 19h, 19n, and 20a had greater activity (MIC ≤ 0.125 *μ*g/mL) than fluconazole (MIC = 0.25 *μ*g/mL). Additionally, the presence of pridinyl group (19a and 19l) 1,2,4-oxadiazole derivatives reduces antifungal activity. On the contrary, compound 19n with furan demonstrated better activity than compound 19b with substitutions on the phenyl ring that revealed distinct effects on antifungal activity. Furthermore, 4-methoxyl (19f), 4-fluoro (19h), and 4-trifluoromethyl (19g) alterations demonstrated promising antifungal activity, with 19g showing the most activity against *C. albicans* (MIC = 0.031 *μ*g/mL). Surprisingly, compound 19c exhibited significant fungicidal activity. In contrast, the antifungal activities of 4-ethyl (19k), 4-chloro (19j), and 4-nitro (19o) derivatives were decreased. On the other hand, fluorine-containing 1,2,4-oxadiazole derivatives such as 20f, 20i, and 20j demonstrated modest antifungal activity. Finally, the heterocyclic pyridinyl derivative 20a demonstrated the greatest activity (Figure 19) [102].

Mahmoudi et al. [103] evaluated some 1,2,4-triazole alcohols bearing *N*-(halobenzyl) piperazine carbodithioate scaffold as effective antifungal agent *in vitro* bioassays versus *C. albicans*, *C*. *glabrata*, *C. parapsilosis*, *C. krusei*, and *C. tropicalis* in which the best activity indicated *N*-(4-chlorobenzyl) derivative 21b with MIC values of 0.063–0.5 mg/mL, being several times more effective than fluconazole. Furthermore, the 3-chlorobenzyl compound 21a displayed a good activity toward both *albicans* and non-*albicans* species of *Candida.* Generally, according to MICs, 2, 4-difluorophenyl derivatives were more active than their dichlorophenyl compounds. In addition, SAR studies revealed that 2,4-difluorophenyl-carbinol was higher than the 2, 4-dichlorophenyl-carbinol scaffold. Moreover, assessment against fluconazole-resistant isolates showed that compound 21b was active against C. *albicans*, *C. krusei*, and *C. parapsilosis* isolates, with MIC values of 2 to 16 mg/mL (Figure 20).

Ciprofloxacin and itraconazole were employed to screen 1,2,4-triazole derivatives fused with novel benzene-ethanol which were assessed at concentrations ranging from 0.125 to 64 mg/mL. Furthermore, compounds 22a, 22g, and 22i showed much better growth inhibitory activity on *C. albicans* with MIC of 32 mg/mL (itraconazole was introduced as the standard drug MIC 1 mg/mL). Electronegativity, like substituent groups on the *para* and *ortho* positions of a benzene ring, can be effective in antifungal activity (Figure 21) [104].

A class of 1,2,4-triazole derivatives has been tested toward *Magnaporthe oryzae*. Aromatic ring structures revealed that the methyl group at position 1,4 of the phenyl ring 23b and the phenyl moiety at the *para* position of phenyl 23c reduced antifungal activity. When an electron-withdrawing fluorine atom entered this position (23e), the antifungal activity increased slightly. An electron-withdrawing group (trifluoromethyl group) had a positive efficacy on increasing the antifungal activity of this synthetic series (comparison of antifungal activity 23b with 23f). The introduction of two chlorine atoms to the phenyl moiety had a distinct effect on increasing antifungal activity. Compound 23g with the 2,4-dichlorophenyl analogue slightly increased the antifungal activity, while compound 23h with the 3,4-dichlorophenyl analogue notably reduced the antifungal activity. The mono chlorine substitution at position 4 of the phenyl ring (23i) reduced the antifungal activity of these synthesized derivatives. According to the preceding considerations, 23e demonstrated remarkable fungicidal activity in this synthetic series. The effect of the chlorine atom on the various positions of the phenoxy moiety (ring B) such as 24a, 24b, and 24c can lead to an increase in antifungal activity. As a result, the fungicidal activity of the analogue without a chlorine substituent at ring B (24j) was the most effective against *M. oryzae* among these compounds (Figure 22) [105].

### 4.2. 1, 2, 4-Triazole Hybrids

Al-Wabli et al. [106] estimated the antifungal characteristics of a variety of novel indole-triazole compounds. The MIC value of compound 25f, which included *N*-phenyl and 3,4-dichlorobenzyl moieties, was 2 mg/mL against *Candida albicans*. In addition, the *para* benzyl substituent exhibits antifungal activity. Also, MIC values for compounds 25b, 25c, 25d, 25e, 25f, and 25g having a phenyl moiety on the triazole ring are 250–500 *μ*g/mL against *Bacillus subtilis*. Meanwhile, compounds 25o, 25p, and 25q with an *N*-cyclohexyl substituent showed moderate to good activity toward the tested *Candida albicans* strain (Figure 23).

The nortopsentin analogues containing 1,2,4-triazole demonstrated good antifungal activity. Compounds 26a, 26d, and 26f were more fungicidal toward *Cercospora arachidicola* Hori than chlorothalonil and carbendazim (commercial fungicides). Compounds 26d and 26f indicated better actions against most of the fourteen plant pathogens (Figure 24) [107].

According to the study by Ahuja et al. [108], compound 27c has a lower ED50 value than the triazole fungicide propiconazole. Significantly, compound 27c showed the highest activity compared with other experimental fungi, with an ED50 value of 16 to 21 *μ*g/mL, which is higher than the ED50 values of the standard commercial fungicides used (tilt: 20–25 *μ*g/mL and carbendazim: 150–230 *μ*g/mL (Figure 25).

Microbiological studies revealed that benzimidazole-1,2,4-triazole hybrid compounds 28m, 28n, 28f, and 28g had good fungicidal activity (MIC50 values of 0.78 to1.56 *μ*g/mL) because of the presence of a fluoro or chloro substituent at the C-*para* position of phenyl, whereas compounds 28c, 28a, and 28b did not. Compounds 28d and 28e demonstrated adequate fungicidal activity (MIC50 values = 1.56–3.12 *μ*g/mL). Compound 28l exhibited comparable antifungal activity with reference drugs fluconazole and ketoconazole. As a result, chloro or fluoro substitution at the C-5 position of benzimidazole is vital and could have had a significant influence on antifungal activity (Figure 26) [109].

The benzimidazole-triazole compounds showed moderate antifungal activity toward *Candida krusei* (ATCC 6258), *Candida glabrata* (ATCC 90030), *Candida albicans* (ATCC 24433), and *Candida parapsilosis* (ATCC 22019), with MIC50 values ranging from 12.5 to 0.78 mg/mL. The findings revealed that compound 3,4-dihydroxy has an influence on the activity (Figure 27) [110].

Novel tri-substituted 1,2,4-triazoles containing benzimidazole were tested for antifungal efficacy against three plant pathogenic fungus, and compounds 30e and 30g showed potent activity against *Venturia nashicola*. However, 30d and 30f indicated sufficient activity against *Fusarium graminearum* (Figure 28) [111].

Luo et al. [112] reported a new group of benzimidazole-derived triazoliums and naphthalimide triazoles that have been thoroughly tested for antifungal activities. Triazoliums 31g and 31f with 3-fluorobenzyl and 2-chlorobenzyl moiety demonstrated the highest antifungal activity (MIC = 2–19 mg/mL) against all tested fungal strains. However, 2,4-di-chlorobenzene triazolium 31h (MIC = 7–29 mg/mL) showed more efficacy than fluconazole (MIC = 7–230 mg/mL). Furthermore, bis (4-fluorobenzyl) triazolium 31b (MIC = 4–19 mg/mL) displayed high activity against all of the microorganisms tested except *S. cerevisiae* (Figure 29).

The antifungal efficacy of 1,2,4-triazoles having quinoline moiety against *A. fumigatus* and *Candida albicans* was highest owing to methoxy and chloro substituents. As a result, 32e, 32g, and 32m derivatives with methoxy and chloro substituents had the highest enhanced activity (Figure 30) [113].

D'Souza et al. [114] investigated the fungicidal of new quinoline-triazoles. Compounds 33b and 34b with chlorine substituents on the aromatic ring demonstrated more antifungal activity than (33e, 33f, 34e, and 34f) that included OCH_3_ and CH_3_ (Figure 31).

Fan et al. [115] investigated the antifungal activity of 1,2,4-triazolo [4,3-a]pyridine-containing quinazoline thioether derivatives at 50 mg/mL. Except for compound 35c against the fungi *Verticillium dahlias* and *Fusarium oxysporum* (inhibition rates of 65.4 and 52.5%, respectively), all of these compounds failed to demonstrate apparent fungicidal activity (≥45%) against the case fungi, with compound 35h against the pathogen *V. dahliae* (46.8%) (Figure 32).

Fan et al. [116] investigated the antifungal activity of quinazolin-containing 1,2,4-triazoles against six significant phytopathogenic fungi in agriculture. Furthermore, compounds 36h and 36g were showed a remarkable fungicidal activity toward *Gloeosporium fructigenum* at 50 mg/mL, comparable to the commercial antifungal hymexazol (Figure 33).

Most of the 2-phenoxy-benzo [*g*] [1, 2, 4] triazolo [1,5-*a*] quinazoline derivatives indicated *in vitro* antifungal activity against ten fungal strains except *C. neoformans.* Nevertheless, 37a and 37b exhibited activity only against *A. niger* and *A. fumigatus*. Compounds 37c, 37d, 37e, 37f, and 38b revealed excellent fungicidal activities against *A. fumigatus* (MIC = 0.98–1.95 *μ*g/mL), and 37g showed the ability to produce amphotericin B (MIC = 0.49 *μ*g/mL). In contrast, 38b had stronger inhibition with respect to the reference drug toward *S. racemosum* (MIC = 0.49 *μ*g/mL) and 37e confirmed similar activities to amphotericin B (MIC = 0.98 *μ*g/mL). In addition, compounds 37c-37e, 38a, and 38b showed the highest activity versus *G. candidum* (MIC = 0.49–0.98 *μ*g/mL) as compared with amphotericin B (MIC = 1.95 *μ*g/mL) (Figure 34) [117].

El-Attar et al. [118] investigated the antifungal activities of 1,2,4-triazolos [4,3-*a*]-quinoxaline derivatives with various substituted pyrazole moieties at position 4. When compared with the reference clotrimazole (MIC = 12.5 *μ*g/mL), compound 39 demonstrated reasonable growth inhibition (MIC = 25 *μ*g/mL) against *C. Albicans*. Compounds 39, 41a, and 41b inhibited only weakly (MIC = 50 *μ*g/mL) growth against the same organism. Clotrimazole activity against the fungus *A. fumigatus* was reduced by one-quarter in studies 39 and 42. Regarding the activity against *R. oryzae*, compounds 39, 40, 41a-c, and 42 showed weak growth inhibition (MIC = 25 *μ*g/mL) when compared with the reference clotrimazole (MIC = 6.25 *μ*g/mL) (Figure 35).

Yang and Bao [119] demonstrated that 1,2,4-triazole derivatives (43a-43k) containing *N*-(substituted phenyl) acetamide and the quinazolinylpiperidinyl moiety group did not exhibit remarkable inhibition activity against phytopathogenic fungi such as *Phytophthora infestans*, *Verticillium dahliae*, and *Gibberella zeae*) at 50 mg/mL save compounds 43e and 43k that showed modest inhibitory activity against the fungus *G. zeae* (Figure 36).

Sompalle et al. [120] investigated the antifungal activity of a class of 1,2,4-triazole-quinazolinethiones (44a-l) against *Aspergillus niger* (*A. niger*) and *Aspergillus flavus* (*A. flavus*) in combination with the commonly used antifungal drug fluconazole (Figure 37).

All triazole derivatives with *N*-alkylated groups were tested for fungicidal activity toward *Candida albicans* and *Aspergillus flavus* and anthelmintic activity against *Pheretima posthuma*, and the compound containing group CH_3_ at the ortho position of the phenyl ring showed good inhibition with the inhibition zone 24.17 ± 0.32 and 15.02 ± 0.41 mm against *A flavus* and *C albicans* in comparison with a standard antifungal drug, Nystatin, while the antifungal activity of the other structures was lower (Figure 38) [121].

Jin et al. [122] investigated the fungicidal activity of novel compounds containing 1,2,4-triazole with different substituted groups toward *Gibberlla nicotiancola*, *Pythium solani*, *Gibberlla saubinetii*, and *Fusarium oxysporum* f.sp*. niveum in vitro*. Compound 46 had good activity against the case fungus, indicating that 1,2,4-triazole-imidazole can contribute to antifungal properties. Methyl at position Q increased the activity, the activity order is 47>46, and compound 47 demonstrated a remarkable antifungal activity. As a result, positions P and Q may have an impact on the activity at the same time (Figure 39).

1,2,4-Triazole derivatives with a pyrimidine moiety were evaluated for fungicidal activity, with compounds 50c and 50d showing the best antifungal activity against *Phompsis* sp. that was even better than pyrimethanil (32.1 mg/mL). Compound 50d, on the other hand, had higher activity against *B. cinerea* and *B. dothidea* with 55.1 and 40.1 mg/mL, respectively, when compared with *Pyrimethanil* (57.6 and 62.8 mg/mL) (Figure 40) [123].

Antifungal evaluation [1, 2, 4] of triazolo [5,1-*b*] quinazolin-8(4*H*) one scaffolds (51a-n) *in vitro* exhibited that compounds 51e and 51i display higher activity than standard drug griseofulvin (MIC 500 mg/mL) against *C. albicans*. Surprisingly, the substitution at the C-6 carbon of the final moiety and *para*-substituted phenyl ring was responsible for variable biological results, while the triazole with nonsubstituted or diversely *para*-substituted (Cl, OCH_3_, and NO_2_) phenyl core or heterocyclic nucleus showed the best properties. In addition, the compounds having OCH_3_ group substitution (compound 51f) effectively showed poor inhibition toward *A. clavatus* and *A. niger* inhibited the *S. aeruginosa*, *P. aeruginosa*, and *S. pneumonia* strains, although the derivative with the electron-withdrawing group such as NO_2_ (compound 51i) efficiently inhibited the *E. coli* bacterial strain as well as was found potent toward the *C. albicans* strain. Finally, compound bearing heteroaryl substitution (compound 51l) led to the improvement in the activity against the *E. coli* strain (Figure 41) [124].

All 1,2,4-triazole having amine derivatives were evaluated and shown to be effective in inhibiting fungal pathogens with MIC values ranging from 1 to 256 *μ*g/mL. They were proposed as the potential antifungal agents that synthesized under optimized conditions as 3(5)-substituted 1,2,4-triazol-5(3)-amine 52. As starting materials, however, several heteroaryl hydrazides and aryls were used as starting materials (Figure 42) [125].

Appna et al. [126] described the fungicidal activity of novel 1,2,4-triazole fused pyrido [2,3-d] pyrimidine derivatives (53a-d and 54a-c) against different *Candida* strains. The antifungal activities of the synthesized compounds 53d, 54b, and 54c were shown. SAR investigations revealed that trifluoromethyl, fluoro, bromo, and nitro groups on the furyl and phenyl rings of *pyrido* [2,3-d] pyrimidine could increase antifungal activity. Compounds (53d, 54b, and 54c) 4-fluoro-2-chlorophenyl triazole and 2-furyl substituent in *pyrido* [2,3-d] pyrimidine exhibited the best activity. As well, 4-nitrophenyl triazole in combination with 2-furyl pyrido [2,3-d] pyrimidine (54b) exhibited the same activity. The antifungal effects of 2-chloro-4-fluoro phenyl triazole with 2-phenyl pyrido [2,3-d] pyrimidine (53d) were favorable (Figure 43).

A new series of 1,2,4-triazole derivatives were synthesized by Singh et al. The antifungal characteristics of the compounds showed that most of them could effectively inhibit the growth of the tested fungal strains. However, none of them were superior to the reference drug fluconazole. Compound 55l had the most potent antifungal activity against both fungi. 55l revealed comparable activity (*A. niger*: MIC = 11.7 *μ*M; *C. albicans*: MIC = 10.9 *μ*M) with the reference fluconazole (*A. niger*: MIC = 9.4 *μ*M; *Candida albicans*: MIC = 10.2 *μ*M). Apart from that, antifungals 55f (*A. niger*: MIC = 15.6 *μ*M; *C. albicans*: MIC = 14.1 *μ*M) and 55a (*A. niger*: MIC = 28.1 *μ*M; *C. albicans*: MIC = 18.8 *μ*M) were found to be potent (Figure 44) [127].

Jin et al. [128] investigated the antifungal effects of a variety of 4-amino-5-substituent-1,2,4-triazole-3-thione Schiff bases toward *Pythium solani*, *Gibberlla nicotiancola*, *Gibberlla saubinetii*, and *Fusarium oxysporum* f.sp. *niveum*. Compounds 56a and 56b showed considerable activity against the majority of the test fungi, while derivative 56a was more potent toward *Gibberlla saubinetii* and *Gibberlla nicotiancola* than triadimefon. The antifungal activity of 56a-d and 57a-d analogues was tested against four plant pathogenic fungi, including *Pythium solani*, *Fusarium oxysporium* f.sp*. niveum*, *Gibberlla nicotiancola*, and *Gibberlla saubinetii* (Figure 45).

Zhang et al. [129] displayed a new class of piperazine-containing 3-(furan-2-yl)-1,2,4-triazole important *in vitro* fungicidal activity toward a variety of plant fungi. In particular, compounds 58a, 58b, 58c, 58d, 58e, 58f, 58g, and 58h showed triadimefon against a variety of test fungi. Compounds 58g, 58f, and 58h having R_1_ = CF_3_ performed better than others (R_1_ = F or Cl). In comparison, the SARs of the compounds revealed 2-positions of the *para* position of substituted benzylideneamino and *ortho* position of phenylpiperazine, where a large group would be favorable for higher fungicidal activity. Finally, compounds with an EWG at the benzyl ring position or an electron-donating group at the 2,4-position of the benzene ring, such as 58b and 58a, demonstrated higher activity (Figure 46).

Trialkylamine compounds having a triazole moiety were evaluated *in vitro* for antifungal activity against six phytopathogenic fungi at 50 mg/mL (*Magnaporthe grisea*, *Curvularia lunata*, *Alternaria solani*, *Fusarium solani*, *A. alternata*, and *F. graminearum*). Compounds 59k (3-F), 59m (3,4-diCl), and 59n (4-Br) had good activity toward *A. solani* with EC50 values of 2.88, 8.20, and 1.92 mg/mL, respectively. Furthermore, compounds 59c (4-Cl), 59f (3,4-diCl), and 59d (2-Br) showed good antifungal activity against *F. graminearum* with EC50 values of 11.60, 5.14, and 16.24 mg/mL, respectively. Also, electron-donating groups 59o (Me) or 59p (OMe) considerably reduced the activity. In contrast, the presence of halogen atoms such as 59k (3-F), 59c (4-Cl), (3,4-diCl), and 59n (4-Br) might increase the activity (Figure 47) [130].

1,2,4-Triazole-pyridine products with hydrazone scaffold (compounds 60a-60h) were tested *in vivo* at 100 mg/mL against *Stemphylium lycopersici* (Enjoji) Yamamoto (SL) and *Fusarium oxysporum* sp. Cucumebrium (FO). Compound 60d as well as compounds having electron-donating groups at the 4-position of benzene such as 60e (*p*-N (CH_3_)_2_), 60b (*p*-F), 60f (*p*- CF_3_), and 60g (*p*-CH_3_) demonstrated strong antifungal activities. As a result, the furan ring-substitution exhibited more activity against SL and FO than the aryl or alkyl groups. Furthermore, both poly- and single-substituted benzene compounds showed excellent activity against FO (Figure 48) [131].

Remarkable antifungal activity of a number of new 1,2,4-triazole derivatives against different strains of *Aspergillus fumigatus*, *Candida albicans*, and *Candida crocus* has been reported in comparison with those of commercial fungicides ketoconazole and itraconazole. All of the derivatives investigated, the dichloro urea analogue and bromo substituted triazole, stand out as the most favorable compounds. The most potent compounds against *A. fumigatus* were 64l, 61b, 61a, and 61c, with MIC values ranging from 0.114 to 0.230 *μ*mol/mL. Instead, amide analogues such as 62f can influence the activity, with the amide moiety 62f having higher activity than less bulky triazoles such as 65o and 65p. Furthermore, compound 63h with the sulfonamide substitution is responsible for the activity reduction. Compounds 64l and 61b have the highest activity, being several times more potent than ketoconazole. Conversely, these derivatives were less active than itraconazole (Figure 49) [132].

Dincel et al. [133] screened a group of novel hydrazinecarbothioamide (66), 4-thiazolidinone (67), and 1,2,4-triazole-3-thione (68) for the fungicidal properties against *C. parapsilosis ATCC 22019*, *C. Albicans ATCC 10231*, *M. gypseum NCPF580*, *C. krusei ATCC 6258*, *T. tonsurans NCPF245*, and *T. mentagrophytes* var. *echinacea*. Generally, 1,2,4-triazole-3-thiones and 4-thiazolidinones showed better fungicidal activity rather than thiosemicarbazide derivatives. As a result, the 3-allyl substitution of 4-thiazolidinones is critical for their antifungal activity. Compounds 67d (R = CH_2_-CH = CH_2_), 68c (R = C_3_H_7_), and 68d (R = CH_2_CH = CH_2_) had the highest fungicidal activity against *S. aureus* (MIC = 32 *μ*g/mL). Also, 68c (R = C_3_H_7_) and 68d (R = CH_2_CH = CH_2_) showed the greatest activity against *E. coli* (MIC = 32 *μ*g/mL). In addition, 68d (R = CH_2_CH = CH_2_) showed the greatest activity towards *P. aeruginosa* (MIC = 32 *μ*g/mL) (Figure 50).

Cheng et al. [134] investigated the fungicidal activity of new groups of 1,2,4-triazole benzoyl aryl amines. The findings revealed a clear relationship between the structure and training in these compounds as well. The electron-withdrawing group *oi*-pr(isopropyl) at the *para* position has a favorable impact on high activity, and the preferred groups were alkoxy carbonyls. This compound indicated the most effective fungicidal activities with EC50 values of 0.12, 0.19, and 0.01 mg/mL against *S. sclerotiorum*, *F. graminearum*, and *G. graminis* var. *tritici*, respectively. Alkoxy carbonyl of these ester carbonyls revealed the highest activities (69a-b and 69c-g). In contrast, no significant increase in the activity was observed when more than one electron-withdrawing group was added to aniline. For instance, if the second electron-withdrawing groups such as CF_3_ or Cl were added to the *meta* situation of aniline, the activity against *G. graminis* var. *tritici* would be reduced (69e and 69f) (Figure 51).

The evaluation indicated that all 1,2,4-triazole derivatives had fungicidal activity, with MIC values ranging from 0.02 to 0.52 mM, which was better than bifonazole (MIC values of 0.32–0.64 mM) and ketoconazole (MIC values of 0.28–1.88 mM). Compound 70c, having a MIC value of 0.02–0.04 mM, exhibited the best antifungal activity rather than compound 70a (Figure 52) [135].

Wu et al. [136] evaluated the fungicidal activity of a novel series of 1,2,4-triazole derivatives containing an amide moiety. Compounds 71a, 71d, 71e, and 71f had the highest antifungal activity against *Botrytis cinerea*. Meanwhile, compound 71b, when R was CH_3_, exhibited better antifungal property against *Phomopsis* sp., compared with that of pyrimethanil. SAR studies revealed that 4-pyridine in the R substituent group and the smaller alkyl substituent groups (H or CH_3_) could have a favorable influence on the activity, such as 71a>71b>71c. Meanwhile, when R = OH is added to the 4-positions of phenyl and substituted phenyl, the action against *Phomopsis* sp., *B. dothidea*, and *B. cinerea* rises in the sequence 71d>71g>71k. Furthermore, when R = 4-pyridine, the antifungal activities of the corresponding compound 71h against *Phomopsis* sp., *B. dothidea*, and *B. cinerea* were higher than those of compound 71e (R = 2-pyridine) (Figure 53).

Yurttaş and CantŘrk [137] investigated triazole-oxadiazole compounds against *C. krusei*, *C. glabrata*, *C. albicans*, and *C. parapsilosis* and found that triazole-oxadiazole derivatives 72e and, particularly, 73i had the highest activity *against C. glabrata* and *C. albicans* (MIC90 = 62.5 mg/mL). The oxadiazole rings of these derivatives differ due to the benzothiazole and phenyl rings linked to the acetamide molecule. Meanwhile, compounds 72e (R = NO_2_) and compound 73e (R = F) were found to have the highest activity (Figure 54).

Li et al. [138] reported a group of *N*-phenylacetamide containing 1,2,4-triazole derivatives (74a-f) that were screened *in vitro* for antifungal assessment, and specific compounds, such as 74b-f derivatives, inhibited the growth of the tested fungus. Among all synthesized compounds, 74a exhibited no antifungal activity. Moreover, mono-substituted halogen substituents in the benzene ring, in either the *ortho* or the *para* position, displayed antifungal activity (Figure 55).

The antifungal properties of the synthesized 1,2,4-triazole-3-yl-mercapto derivatives toward two *Candida albicans* strains (*C. albicans* ATCC 10231 and *C. albicans* ATCC 18804) and one non-*Candida albicans* strain (*C. krusei* ATCC 6258) were evaluated. Its antifungal activity was shown by the presence of a halogenated aryl substituent linked to the 3-mercapto group. Compounds 75d, 75f, and 75g had smaller MIC values than the other 1,2,4-triazolyl-thioethers, indicating that the 1,2,4-triazole-3-yl-mercapto derivatives with a 4-Cl-phenyl component had more excellent antifungal activity against the *Candida krusei* ATCC 6258 strain. In this series, compound 75d in this series has the lowest MIC value (Figure 56) [139].

Antifungal activities of new myrtenal derivatives containing 1,2,4-triazole were tested against *Physalospora piricola*, *Fusarium oxysporum* f.sp. *cucumerinum*, *Cercospora arachidicola*, *Alternaria solani*, and *Gibberella zeae* at 50 mg/mL. Among these compounds, 76a (R = Et), 76c (*R* = i − Pr), and 76e (R = o − NO_2_ Bn) had the most significant antifungal activity against *P*. *piricola*. Among these derivatives, 76a (R = Et) 76c (*R* = i − Pr), and 76e (R = o − NO_2_ Bn) indicated the highest antifungal activity against *P. piricola* (Figure 57) [140].

Cheng et al. [141] evaluated a series of 4,5-disubstituted-3-S-(*β*-D-acetyl glycosyl)-1,2,4-triazoles for their antifungal activities in which compounds revealed reasonable activities at the concentration of 50 *μ*g/mL. Particularly, compounds 77c, 77g, 77n, and 77p displayed 60–68.6% inhibitory rates against *B. cinerea* and 77c, 77d, 77g, 77m, 77n, and 77p derivatives exhibited 63.6%–78.8% inhibitory rates against *S*. *sclerotiorum*, with the antifungal activity of R_2_ = ethyl being lower than those of the other compounds against *S. sclerotiorum*. In other words, compounds containing a galactosyl moiety, such as compound 77n, demonstrated highly favorable antifungal action, whereas compounds with a glucosyl moiety showed comparably weak antifungal activity (Figure 58).

Bitla et al. [142] synthesized and screened *bis*(1,2,3 and 1,2,4)-triazole derivatives for antifungal activity, and compounds 78a, 78d, 78f, and 78i had the highest activity. It is remarked that bromo and chloro substitutes at *meta* and *para* positions of the aryl ring were highly important. Compound 78f indicated superior activity against *S. aureus* MTCC 96 (MIC 3.9 ± 0.05 *μ*g/ml) (Figure 59).

Beyzaei et al. [143] synthesized and tested a new class of 1,2,4-triazole-3-thiones in glycerol/potassium carbonate and assessed them for antifungal activity. Significant inhibitory special effects were detected notably against fungal infections. *Fusarium oxysporum* and *Aspergillus fumigatus* were inhibited with all of them. The most excellent antifungal activities indicated triazole 79c that contains R = 4-nitrophenyl has the highest antifungal activity as well as the high-affinity binding to the receptor. Hydrogen bonds between the *N*-1 azole ring and some amino acid residues in the target enzyme interact predominantly. These findings might aid in the development of antifungal drugs (Figure 60).

Some studies have been conducted on the fungicidal activities of the novel 1,2,4-triazole derivatives. Compounds 80a-d (Figure 61) in particular showed high antifungal activity. The relationship between biological activity and structure revealed that compounds with the sulfur atom exclusively in the thiol form exhibited activity. Furthermore, compounds 80a and 80c, at a concentration of 1000 mm, inhibit the growth of *C. albicans* by 35–40%, respectively [144].

Sidhu and Kukreja [145] reported new compounds based on lead hybridization of 1,2,4-triazoles with fluorinated benzothiazol-2-yl that were tested for fungicidal activity against *P. striiformis*, *D. oryzae*, and *U. hordei* in contrast with conventional fungicides. Furthermore, derivatives 81b and 81c are active against most of the experimental fungi. Compounds 81a and 81e caused the antifungal potential of EC50 0.23 and 0.19 mmoles/L, respectively, against *P. striiformis* that was compared to the standard fungicide (EC50 value 0.10 of mmoles/L). Compound 81a has the greatest EC50 value (0.17 mmoles/L) against *U. hordei* when compared to Vitavax (EC50 value of 0.09 mmoles/L) (Figure 62).

Shingare et al. [146] presented a new series of pyrazole bearing triazolo-thiadiazole derivatives (82a-l) which were evaluated to have antifungal activity versus *A. Niger*, *C. albicans*, and *A. clavatus* along with nystatin and griseofulvin as standard drugs. Amongst them, compounds 82b and 82j revealed good antifungal activity. Compound 82j has shown the most activity (Figure 63).

The antifungal activity of 1,2,4-triazolo containing thiadiazoles (83a-e) and 1,2,4-triazol-3-ylthio-*N*-4-aryl) acetamides (84a-d) was evaluated. Compound 84a had good activity toward *A. flavus* with a MIC value of 70 *μ*g/mL compared with standard fluconazole; derivatives 83d, 83a, 84c, and 84a demonstrated moderate activity (Figure 64) [147].

Bai et al. [148] assessed several novel 1,2,4-triazole analogues for antifungal activity against eight phytopathogens and found that the majority of them exhibited acceptable to outstanding fungicidal characteristics. Almost all of the compounds demonstrated moderate to excellent fungicidal activity toward the tested phytopathogens. In general, the fungicidal activity of methyl oxime ether group 85 (R_1_ = methyl) was significantly greater than benzyl oxime ether group 86 (R_1_ = benzyl). It is clear that electron-drawing groups at the 2-position of the phenyl ring, such as 85b, 85d, 86b were more helpful for fungicidal activity. Because of the halogen substituent effect, compounds 85b, 85d, 85g, 85k, and 86b demonstrated significantly higher inhibitory activities against fungal pathogens than other compounds, with the chlorine atom playing a more significant role in improving fungicidal activity in each position of the benzene ring.

Furthermore, the prevention rates of compounds 85d, 86e, and 85f against all of the fungi examined were meager. It is shown that for benzyl oxime ether series 85, a bulky 2-tert-butyl group on the benzene substituent was not best for the activity. Compound 85d (2-Cl-4-Br) containing two mixed halogen atoms showed broad-spectrum fungicidal activity, with EC50 values of 1.59, 0.46, 0.27, and 11.39 mg/L against four fungal pathogens (Figure 65).

## 5. Conclusion

A privileged structure in medicinal and organic chemistry is 1,2,4-triazole-hybrids having a broad spectrum of antifungal activity. The 1,2,4-triazole nucleus and its derivatives are essential scaffolds in the discovery and development of drugs that have a multitude of biological activities. An acceptable reason for its broad biological profile is a small and stable cyclic ring structure wherein the nitrogen atoms can act both as hydrogen bond donor and as acceptors at the active site of the receptor. The pentacyclic triazole ring processes plasticity for the synthesis of a number of derivatives due to of its multifold binding sites. This potent scaffold will act as a lead molecule in drug synthesis in the future. The various methods for the regioselective synthesis of 1,2,4-triazole-scaffold will be a great tool in medicinal chemistry in the future. The most challenging problem in fungal therapy is antifungal resistance, which may be progressed by drug target overexpression. This review is focused to summarizing recent research on 1,2,4-triazole-hybrids as fungicidal agents over the last decade. It will aid researchers and medicinal chemists in the discovery and the synthesis of new antifungal compounds with 1,2,4-triazole-moiety.

## Figures and Tables

**Figure 1:** Chart related to the content of provided in this review.

**Scheme 1:** Tautomeric forms of the 1,2,4-triazole structure.

**Scheme 2:** The preparation of 1,2,4-triazoles from hydrazines.

**Scheme 3:** Synthesis of 1,2,4-triazole from amidine.

**Scheme 4:** I_2_-mediated oxidative C-N and N-S bond formations.

**Scheme 5:** Synthesis of 1,2,4-triazoles in the presence of Cu (II) catalysis.

**Scheme 6:** The synthesis of 1,2,4-triazoles of hydrazones and aliphatic amines.

**Scheme 7:** Arylation reactions of 1,2,4-triazoles.

**Scheme 8:** Alkylation reactions of 1,2,4-triazoles.

**Scheme 9:** Direct synthesis of *N*4-substituted triazoles.

**Figure 2:** Chemical structures of some bioactive 1,2,4-triazole-based marketed drugs.

**Figure 3:** Structure-activity relationship of fluconazole.

**Figure 4:** The structure of 1, 2, 3-benzotriazin-4-one.

**Figure 5:** Antifungal screening of novel hybrids of triazole derivatives.

**Figure 6:** Chemical structure of novel azole antifungals containing a fused triazinone scaffold.

**Figure 7:** Chemical structure of novel triazole analogues featuring isoxazole moieties.

**Figure 8:** Novel triazole derivatives bearing alkynyl side chains.

**Figure 9:** Benzylthio analogues of fluconazole.

**Figure 10:** The study of antifungal properties in new fluconazole derivatives.

**Figure 11:** Structure of azoles containing imidazole derivatives.

**Figure 12:** Antifungal assessment of new triazole derivatives.

**Figure 13:** Fluconazole-derivatives bearing nitrotriazol or 2-(piperazine-1-*y*lFig) ethanol moieties.

**Figure 14:** New triazole derivatives of ravuconazole and isavuconazole.

**Figure 15:** Structure of triazole-piperdine-heterocycle.

**Figure 16:** Structure of novel t hybrids of 5-flucytosine and fluconazole.

**Figure 17:** Novel triazole derivatives bearing *γ*-lactam.

**Figure 18:** Structure-activity relationship between triazoles as miconazole analogues.

**Figure 19:** Structure-activity relationship between triazoles bearing piperdine-oxadiazoleside chains.

**Figure 20:** Triazole alcohols holding *N*-benzylpiperazine carbodithioate moiety.

**Figure 21:** Novel benzene-ethanol bearing 1,2,4-triazole derivatives.

**Figure 22:** 1-(4-Phenoxymethyl-2-phenyl-[1, 3] dioxolan-2-ylmethyl)-1*H*-1,2,4-triazole derivatives.

**Figure 23:** Evaluation of the antifungal activity of new indole-1,2,4-triazole conjugates.

**Figure 24:** 1,2,4-Triazole derivatives containing nortopsentin.

**Figure 25:** Benzimidazolyl-1,2,4-triazole.

**Figure 26:** SAR outline of the benzimidazole-1,2,4-triazole hybrid compounds.

**Figure 27:** Structure of new benzimidazole-triazoles.

**Figure 28:** Tri-substituted 1,2,4-triazoles containing benzimidazole moiety.

**Figure 29:** Structure-activity relationships between benzimidazole-derived naphthalimide triazoles.

**Figure 30:** 1,2,4-Triazole hybrids of 2-(aryloxy) quinolones.

**Figure 31:** Antifungal activity evaluation of quinolone-triazole derivatives.

**Figure 32:** Quinazoline thioether-1,2,4-triazolo [4,3-a] pyridine derivatives.

**Figure 33:** 1,2,4-Triazole containing quinazolin derivatives.

**Figure 34:** Chemical structure of 2-phenoxy-benzo-triazole quinazoline derivatives.

**Figure 35:** Antifungal study on pyrazol-1,2,4-triazol-quinoxalines.

**Figure 36:** 1,2,4-Triazole derivatives containing the quinazolinylpiperidinyl moiety.

**Figure 37:** SAR study of triazolo-quinazolinethiones.

**Figure 38:** Structure of triazole derivatives containing *N*-alkylation.

**Figure 39:** Chemical structure of novel 1,2,4-triazole derivatives.

**Figure 40:** The structure of triazole derivatives with a pyrimidine moiety.

**Figure 41:** [1, 2, 4] Triazolo [5,1-*b*] quinazolin-8(4*H*) derivatives.

**Figure 42:** Study of 1,2,4-triazole derivatives.

**Figure 43:** Chemical structure of new 4-hydrazone functionalized/1,2,4-triazole fused pyrido [2,3-d] pyrimidine derivatives.

**Figure 44:** Antifungal evaluation of novel bioactive 1,2,4-triazoles.

**Figure 45:** Chemical structure of new 1,2,4-triazole Schiff base derivatives.

**Figure 46:** Study of the structure of new piperazine-bearing 3-(furan-2-*y*l)-1, 2, 4-triazole.

**Figure 47:** Structure of trialkylamine derivatives bearing a triazole moiety.

**Figure 48:** (SAR) analysis of 1,2,4-triazolo-pyridine derivatives containing hydrazone moiety.

**Figure 49:** The study of antifungal properties of 1,2,4-triazoles.

**Figure 50:** Structure of hydrazinecarbothioamides, 4-thiazolidinones, and 1,2,4-triazole-3-thiones.

**Figure 51:** The structure of 1,2,4-triazole benzoyl arylamine compounds.

**Figure 52:** New vinyl-1, 2, 4-triazole analogues.

**Figure 53:** 1,2,4-Triazole derivatives bearing an amide moiety.

**Figure 54:** The study of some triazole-oxadiazole compounds.

**Figure 55:** The study of *N*-phenylacetamide containing 1,2,4-triazole derivatives.

**Figure 56:** The chemical structures of 1, 2, 4-triazole-3-yl-mercapto derivatives.

**Figure 57:** Novel myrtenal-based 4-methyl-1, 2, 4-triazole-thioethers.

**Figure 58:** 1,2,4-Triazole with glucosyl moiety compounds.

**Figure 59:** Assessment of *bis*-1,2,4-triazole derivatives as antifungal agents.

**Figure 60:** Antifungal study on 4,5-substituted 1,2,4-triazole-3-thiones.

**Figure 61:** Derivatives of 1,2,4-triazole with a thiomethyl bridge.

**Figure 62:** Series of new fluorinated benzothiazol-2-yl-1,2,4-triazoles.

**Figure 63:** Chemical structures of pyrazole bearing triazolo-thiadiazole derivatives.

**Figure 64:** The study of the chemical structure of triazole based heterocycles.

**Figure 65:** 1,2,4-Triazole analogues having oxime ether and phenoxyl pyridinyl moiety.

**Table 1:** Pharmacological properties and clinical implications of all marketing antifungal drugs.

Drug/PubChem ID	Chemical name	Action of antifungal	Ref.
Itraconazole, CID: 55283	2-Butan-2-yl-4-[4-[4-[4-[[(2R,4S)-2-(2,4-dichlorophenyl)-2-(1,2,4-triazol-1-ylmethyl)-1,3-dioxolan-4-yl]methoxy]phenyl]piperazin-1-yl]phenyl]-1,2,4-triazol-3-on	Treatment of *onychomycosis* and *seborrheic* dermatitis	[51–53]
Fluconazole, CID: 3365	2-(2,4-Difluorophenyl)-1,3-bis(1*H*-1,2,4-triazol-1-yl)propan-2-ol	Effect on *blastomycosis*, *cryptococcosis*, *candidiasis*, *coccidioidomycosis*, *histoplasmosis*, *dermatophytosis*, and *pityriasis* versicolor	[54, 55]
Isavuconazole, CID: 6918485	4-[2-[(2*R*,3R)-3-(2,5-Difluorophenyl)-3-hydroxy-4-(1,2,4-triazol-1-yl) butan-2-yl]-1,3-thiazol-4-yl] benzonitrile	To treat invasive *aspergillosis* and invasive *mucormycosis*	[56, 57]
Efinaconazole, CID: 489181	(2*R*, 3R)-2-(2, 4-Difluorophenyl)-3-(4-methylidenepiperidin-1-yl)-1-(1, 2, 4-triazol-1-yl) butan-2-ol	The treatment of *onychomycosis* (nail fungal infection)	[58–60]
Posaconazole, CID: 468595	4-[4-[4-[4-[[(3*R*,5*R*)-5-(2,4-Difluorophenyl)-5-(1,2,4-triazol-1-ylmethyl)oxolan-3-yl]methoxy]phenyl]piperazin-1-yl]phenyl]-2-[(2*S*,3*S*)-2-hydroxypentan-3-yl]-1,2,4-triazol-3-one	For the treatment of *aspergillus* and *Candida* and invasive fungal infections caused by the treatment of *Scedosporium* and *fusarium* species of pharyngeal *candidiasis* (OPC), including OPC retrofitting in the treatment of itraconazole and/or fluconazole	[61–66]
Voriconazole, CID: 71616	(2*R*, 3S)-2-(2, 4-Difluorophenyl)-3-(5-fluoropyrimidin-4-yl)-1-(1, 2, 4-triazol-1-yl) butan-2-ol	Treatment includes *candidiasis*, *coccidioidomycosis*, *histoplasmosis*, *penicilliosis*, *aspergillosis*, and infections by *Scedosporium* or *fusarium*	[67–70]
Albaconazole, CID: 208952	7-Chloro-3-[(2*R*, 3R)-3-(2, 4-difluorophenyl)-3-hydroxy-4-(1, 2, 4-triazol-1-yl) butan-2-yl] quinazolin-4-one	Treatment of antiprotozoal agent	[71]
Ravuconazole, CID: 467825	4-[2-[(2R, 3R)-3-(2, 4-Difluorophenyl)-3-hydroxy-4-(1, 2, 4-triazol-1-yl) butan-2-yl]-1, 3-thiazol-4-yl] benzonitrile	Limited activity against species of *Scedosporium*, *fusarium*, and *zygomycetes*	[72–74]
Propiconazole, CID: 43234	1-[[2-(2,4-Dichlorophenyl)-4-propyl-1,3-dioxolan-2-yl]methyl]-1,2,4-triazole	In terms of agriculture as a systemic fungicide grown in meadow plants for seeds and aesthetic value, sports, wheat, mushrooms, corn, wild rice, peanuts, almonds, sorghum, oats, pecans, apricots, peaches, nectarines, plums, and prunes are used	[75, 76]
Fosravuconazole, CID: 9807507	[(2R,3R)-3-[4-(4-Cyanophenyl)-1,3-thiazol-2-yl]-2-(2,4-difluorophenyl)-1-(1,2,4-triazol-1-yl)butan-2-yl]oxymethyl dihydrogen phosphate	Treatment of *onychomycosis*, fungal nail infections, and treatment of *eumycetoma*	[31, 77]
Fosfluconazole, CID: 214356	{[2-(2,4-Difluorophenyl)-1,3-bis(1*H*-1,2,4triazole-1-yl)propan-2-yl]oxy}cphosphonic acid	Treatment and prevention of superficial and systemic fungal infections	[78]
Flusilazole, CID: 73675	1-{[Bis(4-fluorophenyl)methylsilyl]methyl}-1*H*-1,2,4-triazole	Used to control fungal infections in a variety of fruit and vegetable products	[79–81]
Tebuconazole, CID: 86102	(RS)-1-(4-Chlorophenyl)-4,4-dimethyl-3-(1*H*, 1,2,4-triazol-1-ylmethyl)pentan-3-ol	Used in agriculture to treat pathogenic fungi of plants	[82]
Triadimefon, CID: 39385	1-(4-Chlorophenoxy)-3,3-dimethyl-1-(1*H*-1,2,4-triazol-1-yl)butan-2-one	Used in agriculture to control various fungal diseases	[83]
Metconazole, CID: 86210	5-[(4-Chlorophenyl)methyl]-2,2-dimethyl-1-(1,2,4-triazol-1-ylmethyl)cyclopentan-1-ol	To control a wide range of fungal infections including *Alternaria*, *rust*, *fusarium*, and *Septoria*	[84]
Paclobutrazol, CID: 158076	(2RS,3RS)-1-(4-Chlorophenyl)-4,4-dimethyl-2-(1,2,4-triazol-1-yl)pentan-3-ol	Plant growth inhibitor, triazole fungicide, root growth, and drought stress resistance can be used as a chemical method to reduce the risk of habitat in cereal crops	[85]
Myclobutanil, CID: 6336	2-(4-Chlorophenyl)-2-(1,2,4-triazol-1-ylmethyl)hexanenitrile	Used as a fungicide which is a steroid demethylation inhibitor, specially inhibiting ergosterol biosynthesis	[86, 87]

## Data Availability

The datasets used and analyzed during the current study are available from the corresponding author on reasonable request. We have presented all data in the form of figures.

## Abbreviations

*A. flavus*: *Aspergillus flavus*
*A. niger*: *Aspergillus niger*
*C. albicans*: *Candida albicans*
C_2_H_3_N_3_: Molecular formula of 1,2,4-triazole derivatives
CuO: Copper (II) oxide or cupric oxide
CYP51: Lanosterol 14*α*-demethylase
ED50: Effective dose for 50% of the population
EWG: Electron withdrawing group
FLC: Fluconazole
FO: Fusarium oxysporum
K_3_PO_4_: Tripotassium phosphate
MIC: Minimum inhibitory concentration
NaOH: Sodium hydroxide
SAR: Structure-activity relationship
SL: *Stemphylium lycopersici*.
